The article "Research on the Relationship Model between Professional Identity and Life Meaning of Clinical Medical Freshmen based on Artificial Intelligence Medical Image Detection" was published in 2022. Journal: Contrast Media Mol Imaging.

# Research on the Relationship Model between Professional Identity and Life Meaning of Clinical Medical Freshmen based on Artificial Intelligence Medical Image Detection

**DOI:** 10.1155/2022/2798513

**Published:** 2022-06-29

**Authors:** Xiufeng Li, Ping Li, Yaxuan Gao, Tan Wang, Ying He, Xinhui Li

**Affiliations:** ^1^Department of Nursing, School of Medicine, Shihezi University, Shihezi City 832000, China; ^2^Department of Public Health and Preventive Medicine, School of Medicine, Shihezi University, Shihezi City 832000, China

## Abstract

**Objective:**

To understand the current situation of professional identity and life significance of clinical medical freshmen in a university in Xinjiang, analyze its influencing factors, find out the influencing factors and causes, and intervene and improve them. Provide the public with better medical and health management services, so that people can independently and effectively predict and prevent diseases; at the same time, it can also guide people to make more correct and wise choices in uncomfortable situations.

**Methods:**

A questionnaire survey was conducted on 793 freshmen majoring in clinical medicine with the college students' professional identity questionnaire and the Chinese version of the meaning in life scale (C-MLQ).

**Results:**

The freshmen total score of professional identity was (97.48 ± 12.21). The total score of meaning in life was (53.26 ± 7.15), and the meaning in life and the professional identity were significantly positively correlated (*r* = 0.467, *P* < 0.01). Students with first choice, only child, urban living, and parents with a high educational level scored higher in their professional identity (*P* < 0.05). First choice (*β* = −0.11, *P* < 0.001), place of residence (*β* = −0.07, *P*=0.03), father's education level (*β* = 0.08, *P*=0.04), family monthly income (*β* = −0.09, *P*=0.02), and the presence of meaning in life (*β* = 0.54, *P* < 0.001) are the influencing factors of students' professional identity. Both professional identity and meaning in life have important relationship with the mental health of medical students. In the development of modern medicine, finding personal career orientation and goals helps to establish a correct outlook on life, values, and the world. It has a positive impact on the development of personal physical and mental health.

**Conclusion:**

The professional identity and life meaning of clinical medical freshmen are at the upper middle level, which can be improved through medical education and other measures. The joint efforts of society, schools, families, and individual students are needed to improve the professional identity of medical students.

The article "Research on the Relationship Model between Professional Identity and Life Meaning of Clinical Medical Freshmen based on Artificial Intelligence Medical Image Detection" was published in 2022. Journal: Contrast Media Mol Imaging.

## 1. Introduction

In the development of medical technology in the modern society, how to train the next generation of doctors within the existing medical resources is the primary consideration. It is an important content to cultivate the professional identity of active medical students. Gleeson A doctor's professional identity is how he perceives and conducts himself as a doctor and as such is a complex structure that connects motivations and competencies to acceptable professional roles [1]. Forouzadeh et al. There is a reciprocal relationship between the formation of a desirable professional identity and the development and strengthening of professionalism [2]. Monrouxe et al. A longitudinal cohort study conducted on the junior doctors, which is a critical period of transition from medical students to professional doctors, suggested that professional identity was significantly negatively related to burnout, including personal and work-related burnout [3]. Ji et al. research found that professional identity has a significant negative predictive effect on college students' depression, and professional identity has a “boiled frog” effect on college students' depression [4]. Zhang and Li In addition, professional identity also has an important impact on learning motivation and learning engagement [5, 6]. Therefore, the study of medical students' professional identity and life significance has certain reference and predictive significance for improving doctors' professional awareness and can provide a certain basis for early intervention. In addition, understanding the professional identity of medical students can discover their potential psychological problems in advance and carry out preventive intervention and timely treatment. King et al. The meaning of life refers to the subjective feeling and experience of meaningful life [7]. Lin It can make people feel that their life is meaningful, beyond the ordinary, and that they have a clear purpose, mission, or overall goal [8]. Czekierda et al. The study found that the meaning of life is related to physical and mental health. As long as we can live actively, it is also a kind of respect for life. It is also a good performance. Mental health is very important to life. Only when you can get healthy mentally and physically can you continue your life and give full play to the meaning of life [9]. It can alleviate anxiety, regulate stress, and play an important role in coping with diseases. In addition, the meaning of life is a predictor of the overall health status of medical students [10].

In view of this, this study investigated the status quo of clinical medical freshmen's professional identity and meaning in life, analyzed the influencing factors of professional identity, and provided intervention directions for improving medical students' professional identity, promoting their mental health.

The article "Research on the Relationship Model between Professional Identity and Life Meaning of Clinical Medical Freshmen based on Artificial Intelligence Medical Image Detection" was published in 2022. Journal: Contrast Media Mol Imaging.

## 2. Methods

### 2.1. Study Design and Participants

Using the method of cluster sampling, in October 2020, 793 freshmen majoring in clinical medicine in a university in Xinjiang were selected as the research objects. Inclusion criteria were freshmen in clinical medicine from a university in Xinjiang; those who gave informed consent and voluntarily participated in the survey. Exclusion criteria were those who have experienced major life events recently; those who are unwilling to participate in this survey.

An online survey platform (https://www.wjx.cn) in China was used in this study. We contacted the head teacher of students and invited them to send the online questionnaire to their students. Students enter the platform by scanning the code to answer the online questionnaire. Before the questionnaire survey, the purpose, significance, and precautions of this study were explained to the students, and the test was administered after the informed consent of the students was obtained. Questionnaire exclusion criteria were answering time is too short (<2 min); answer options are consistent.

The telephone interview questionnaire is easier to understand. It is to explain the purpose of the research to the respondents and ask questions in the form of telephone communication. The questioner shall fill in the questions according to the answers of the respondents on the phone.

### 2.2. Measure

#### 2.2.1. Demographic Characteristics

Demographic factors include age, gender, nationality, political status, whether to serve as a class cadre, whether clinical medicine is their first choice, whether they are the only child in their family, family residence, parental education level, parental occupation, and family monthly income. Demography is more prominent in population growth strategy analysis, population aging analysis, fertility analysis, mortality and life expectancy analysis, population migration and urbanization analysis, family and marriage analysis, demographic data evaluation, etc.

#### 2.2.2. Professional Identity

The Professional Identity Questionnaire for Undergraduate Students (PIQUS) was compiled in a Chinese language by Qin to measure professional identity among the undergraduate students [11]. This instrument contains 23 items and yields scores on the following four dimensions: cognition (five items), emotionality (eight items), behavior (six items), and fitness (four items). Items are accessed on a 5-point Likert scale (“complete conformity”= 5, “conformity”= 4, “neutral”= 3, “inconformity”= 2, and “complete inconformity”= 1). The reliability of this scale was confirmed with Cronbach's alpha coefficient of 0.95. The total scores are calculated by the sum of scores of each question divided by the total number of questions; high scores indicate high level of professional identity.

The article "Research on the Relationship Model between Professional Identity and Life Meaning of Clinical Medical Freshmen based on Artificial Intelligence Medical Image Detection" was published in 2022. Journal: Contrast Media Mol Imaging.

#### 2.2.3. Meaning in Life

The meaning in life was measured by the 10-item Chinese version of the Meaning in Life Scale (C-MLQ) [12]. It included two dimensions: the presence of meaning in life (5 items), the search for meaning in life (5 items), and using a 7-point scale (1= not true at all; 7= totally true). The reliability of this scale's two dimensions was confirmed with Cronbach's alpha coefficient of 0.85 and 0.82, respectively. The higher the score, the stronger the sense of meaning in life.

#### 2.2.4. Data Analysis

SPSS 20.0 was used for statistical analysis of data. Statistical descriptions are expressed as the mean ± standard deviation. The Pearson correlation was used to analyze the relationship between the meaning in life and the professional identity. The independent *t*-test and one-way analysis of variance (ANOVA) were used to test whether there were differences in the scores of students' professional identity among different groups, multiple linear regression was used to test the influencing factors of clinical medical freshmen's professional identity, and the test level was *P* < 0.05.

## 3. Results

### 3.1. Demographic Characteristics

In this study, a total of 793 questionnaires were distributed, 781 questionnaires were returned, and 8 invalid questionnaires were excluded. Finally, 773 valid questionnaires remained, with an effective rate of 97.48%. Most of the respondents were aged 18–20; there were 353 boys and 420 girls, with a male-to-female ratio of 0.84:1; 78.90% of the students were first-choice students, and only 21.10% were transfer students; the only child accounted for 66.10%; 483 students were urban residents, and 290 students were from rural areas; only 24 fathers and 35 mothers were medical staff, and the rest of the students' parents were nonmedical staff; most of the parents had primary and junior high school education; 64.55% of students have a monthly household income of 3000–10000, and only a small number of families have a monthly income of less than 3000 (194 students) or more than 10000 (80 students).

### 3.2. The Score of the Professional Identity of Freshmen in Clinical Medicine

The total score of students' professional identity was (97.48 ± 12.21), and the item average score was 4.24, which was higher than the intermediate critical value (3). Overall, students had above-average levels of professional identity, with scores above the median cutoff for all four dimensions (Table 1).

The article "Research on the Relationship Model between Professional Identity and Life Meaning of Clinical Medical Freshmen based on Artificial Intelligence Medical Image Detection" was published in 2022. Journal: Contrast Media Mol Imaging.

### 3.3. The Score of the Meaning in Life of Freshmen in Clinical Medicine

The total score of the meaning in life of students was (53.26 ± 7.15), the average score of the items was 5.33, which was higher than the intermediate critical value (4), and the scores of both dimensions were higher than the intermediate critical value (Table 2).

### 3.4. Correlation Analysis between the Meaning in Life and the Professional Identity of Freshmen in Clinical Medicine

The Pearson correlation analysis was performed on the total score and the 2 subdimensions scores of meaning in life and the total score and the 4 dimension scores of professional identity. The results showed that there was a significant positive correlation between the meaning in life and the professional identity (*r* = 0.467, *P* < 0.01). Each dimension of the meaning in life was positively correlated with each dimension of professional identity, and the correlation coefficient was 0.165–0.576 (Table 3).

### 3.5. Univariate Analysis on the Professional Identity of Freshmen in Clinical Medicine

The results of the comparison between different groups show that the total score and the scores of each dimension of professional identity are different between the first choice and the nonfirst choice, the only child and the nononly child, the urban and the rural, the different parental education levels, and the differences are statistically significant (*P* < 0.05) (Table 4).

### 3.6. Multivariate Analysis of the Professional Identity of Freshmen in Clinical Medicine

Taking the total score of students' professional identity as the dependent variable and the significant variable in the univariate analysis as the independent variable, the multiple linear regression analysis was carried out. The regression model is meaningful, *F* = 35.19 (*P* < 0.001), the tolerance is greater than 0.1, the VIF is less than 10, there is no multicollinearity between the data, and the residuals are approximately normal distribution. The results of linear regression analysis showed that whether or not the first choice (*β* = −0.11, *P* < 0.001), place of residence (*β* = −0.07, *P*=0.03), father's educational level (*β* = 0.08, *P*=0.04), family monthly income (*β* = −0.09, *P*=0.02), and the score of the presence of a meaning in life (*β* = 0.54, *P* < 0.001) were the influencing factors of the professional identity of freshmen in clinical medicine (*P* < 0.05) (Table 5).

## 4. Discussion

The professional identity of clinical medical freshmen is at the upper middle level, which can be improved by carrying out medical education and other measures to enhance the professional responsibility and learning interest of medical students, strengthen the service awareness, and improve the professional identity through the combination of theory and practice.

The article "Research on the Relationship Model between Professional Identity and Life Meaning of Clinical Medical Freshmen based on Artificial Intelligence Medical Image Detection" was published in 2022. Journal: Contrast Media Mol Imaging.

The professional identity score in this study is higher than that in previous studies [11, 13]. It shows that the freshmen of clinical medicine have a high degree of recognition of their majors. The scores of each dimension are emotionality >behavior >cognition >fitness, which is consistent with the findings of Zhou et al. [14], and the emotional professional identification score is the highest, indicating that students recognize this major psychologically and emotionally. The fitness professional identity score is the lowest, indicating that students should improve their own adaptability and ability to resist pressure and continuously improve their own suitability. One study shows that COVID-19 has positive effects on students' professional identity [15]. The freshmen in this study were all enrolled after the epidemic. The background of the epidemic and the students' own experiences may lead to higher levels of students' professional identity than other studies.

### 4.1. The Life, Meaning of Life, and Mental Health Problems of Clinical Medicine Freshmen at the Upper-Middle Level

The meaning of life is related to mental health. Only when we understand our own value of life can we better pursue the meaning of life. People with a meaningful life are usually more satisfied with life than those without a meaningful life. Only when we pursue life can our hearts be stronger [16]. This study is consistent with the findings of Ji and Zang [17], and the overall level of the meaning of life for freshmen in clinical medicine is relatively high. The subdimension scores are the presence of meaning in life >the search for meaning in life. It shows that the freshman's current experience and perception of his life are very meaningful, but the degree of enthusiasm for searching the meaning or goal of life still needs to be improved.

### 4.2. The Meaning in Life Is an Important Predictor of the Professional Identity of Freshmen in Clinical Medicine

The results of this study showed that there was a significant positive correlation between the meaning in life and the professional identity of freshmen in clinical medicine (*P* < 0.01). This indicated that the higher the student's sense of meaning in life, the higher the professional identity. Undergraduate students are in the early stage of youth, a crucial period for personality development and ego identity, and they have the will to actively pursue the meaning in life [18]. People who have found their meaning in life are psychologically healthier and adapt better socially [19, 20]. In contrast, people with a lower meaning of life are more likely to be lonely [21, 22], anxious, and depressed [23]. Research shows that students with a strong sense of meaning in life have significantly higher professional identity than students with a low sense of meaning in life, and the strength of the sense of meaning in life has an important impact on students' professional identity [24]. Zhu and Yao research shows that the existence of high-level life significance plays an important role in reducing depression [25]. Identifying with yourself or an important object closely related to yourself can significantly reduce the level of depression [26]. In view of this, schools should pay more attention to the relationship between the meaning of life and the professional identity, guide students to find meaningful life goals, enhance their professional identity, and reduce the risk of psychological problems of medical students.

The article "Research on the Relationship Model between Professional Identity and Life Meaning of Clinical Medical Freshmen based on Artificial Intelligence Medical Image Detection" was published in 2022. Journal: Contrast Media Mol Imaging.

### 4.3. The Professional Identity of Freshmen in Clinical Medicine Is Affected by Multiple Factors

The reason for major choice is one of the factors that affect students' professional identity, and the first-choice students generally have a higher professional identity. The students who selected the major due to personal interests showed a higher level of professional identity than the students who enrolled in the major because of recommendations of family members or teachers [27]. Therefore, teachers and parents should fully respect the decisions of students and provide guidance based on the personality traits and interests of students.

Residence is another factor influencing students' professional identity. The results show that the professional identity of urban students is higher than that of rural students. Affected by the environment, the living standard and medical treatment level in rural areas are average than in urban areas, which is not conducive to the psychological acceptance of medical students. It is one of the negative factors that affect the professional identity. It is suggested that schools should pay attention to the improvement of the medical professional identity of rural students, deepen the understanding of the clinical medical profession, and promote the suitability of themselves and medicine.

The educational level of the father is in direct proportion to the vocational identity of the students. The higher the educational level of the parents, the higher the recognition of the children in vocational certification. Students of the Canadian English medical college are more likely to have grown up in high-income families. Their parents are professionals with a high level of formal education. They instill influence on their children's education from an early age and have a high degree of recognition for their professional identity [28]. This has something to do with parents' understanding of the medical profession and the employment guidance they can provide. The higher the father's education level, the more professional guidance he provides to his children, and the higher the student's recognition of the selected major. This also reflects that the improvement of students' professional identity also needs the participation of families.

The article "Research on the Relationship Model between Professional Identity and Life Meaning of Clinical Medical Freshmen based on Artificial Intelligence Medical Image Detection" was published in 2022. Journal: Contrast Media Mol Imaging.

Family monthly income is inversely proportional to students' professional identity, similar to a foreign research [29], indicating that students with a high monthly family income have a weaker professional identity, which is related to the fact that children from wealthy families may give priority to majors with high income and a comfortable working environment. The working environment of doctors is relatively complex, and the contradiction between doctors and patients in China always exists, so students from high-income families have low professional recognition of clinical medicine.

## 5. Conclusions

To sum up, the professional identity and meaning in life of freshmen in clinical medicine are at the upper-middle level. Both of them have an important relationship with the mental health of medical students. Therefore, the school should strengthen the intervention on the meaning of life and professional identity of medical students, carry out a good combination of learning, training, education, and practice, pay attention to the psychological education of medical freshmen, guide students to find meaningful life goals, enhance their professional identity, and then promote the mental health of medical students. Besides, the improvement of medical students' professional identity requires the joint efforts of society, schools, families, and individual students. The profession of medical students is closely related to the society. It plays a connecting role in the further development of the medical field in China. It is the basis for training the next generation of medical talents. They will not fade with the changes of the times. On the contrary, with the increasing professionalization of medical students in social problems, the socialization of medical problems is becoming more and more prominent, resulting in a closer relationship between medicine and society.

## Figures and Tables

**Table 1:** Professional identity scores of freshmen in clinical medicine (*n* = 773).

	Dimension scores	Item average scores
Cognition	21.74 ± 2.66	4.35 ± 0.53
Emotionality	35.30 ± 4.65	4.41 ± 0.58
Behavior	24.91 ± 3.72	4.15 ± 0.62
Fitness	15.53 ± 2.91	3.88 ± 0.73

The article "Research on the Relationship Model between Professional Identity and Life Meaning of Clinical Medical Freshmen based on Artificial Intelligence Medical Image Detection" was published in 2022. Journal: Contrast Media Mol Imaging.

**Table 2:** Scores on the meaning in life for freshmen in clinical medicine (*n* = 773).

	Dimension scores	Item average scores
The presence of meaning in life	26.81 ± 4.13	5.36 ± 0.93
The search for meaning in life	26.46 ± 4.67	5.29 ± 0.72
Total scores	53.26 ± 7.15	5.33 ± 0.79

**Table 3:** Correlation analysis between the meaning in life and the professional identity (*r* value).

Dimension	Cognition	Emotionality	Behavior	Fitness	Total scores
The presence of meaning in life	0.462 ^*∗*^ ^*∗*^	0.435 ^*∗*^ ^*∗*^	0.568 ^*∗*^ ^*∗*^	0.571 ^*∗*^ ^*∗*^	0.576 ^*∗*^ ^*∗*^
The search for meaning in life	0.165 ^*∗*^ ^*∗*^	0.166 ^*∗*^ ^*∗*^	0.192 ^*∗*^ ^*∗*^	0.201 ^*∗*^ ^*∗*^	0.206 ^*∗*^ ^*∗*^
Total scores	0.375 ^*∗*^ ^*∗*^	0.360 ^*∗*^ ^*∗*^	0.454 ^*∗*^ ^*∗*^	0.461 ^*∗*^ ^*∗*^	0.467 ^*∗*^ ^*∗*^

*Note.* ^*∗*^ ^*∗*^*P* < 0.01

**Table 4:** Comparison of professional identity scores between different groups (*n* = 773).

Variable		N	Cognition	Emotionality	Behavior	Fitness	Total scores
Age	≤18 years	392	21.76 ± 2.53	35.16 ± 4.67	24.78 ± 3.63	15.48 ± 2.80	97.18 ± 11.95
	>18 years	381	21.72 ± 2.79	35.45 ± 4.64	25.05 ± 3.82	15.58 ± 3.02	97.80 ± 12.48

*t*			0.23	0.86	−1.03	0.46	0.70
*P*			0.82	0.39	0.30	0.65	0.48
Gender	Male	353	21.78 ± 2.94	35.10 ± 5.01	24.89 ± 4.15	15.83 ± 3.02	97.60 ± 13.45
	Female	420	21.70 ± 2.40	35.47 ± 4.32	24.93 ± 3.33	15.28 ± 2.79	97.38 ± 11.07

*t*			0.44	−1.09	0.15	2.60	0.25
*P*			0.66	0.28	0.88	0.01^*∗*^	0.80
Nationality	Han nationality	632	21.68 ± 2.74	35.10 ± 4.76	24.79 ± 3.85	15.46 ± 2.96	97.03 ± 12.59
	Minority	141	21.99 ± 2.78	35.18 ± 4.04	25.45 ± 3.07	15.87 ± 2.68	99.50 ± 10.16

*t*			−1.26	−2.51	−1.91	−1.51	−2.17
*P*			0.21	0.01^*∗*^	0.06	0.13	0.03^*∗*^
Political status	Communist youth league	673	21.75 ± 2.68	35.35 ± 1.64	24.89 ± 3.76	15.47 ± 2.93	97.47 ± 12.26
	Other	100	21.61 ± 2.55	34.91 ± 4.75	24.99 ± 3.45	15.88 ± 2.70	97.38 ± 11.90

*t*			0.51	0.88	−0.24	−1.29	0.07
*P*			0.61	0.38	0.81	0.20	0.94
Class cadre	Yes	413	21.78 ± 2.65	35.37 ± 4.77	24.87 ± 3.83	15.52 ± 3.06	97.53 ± 12.57
	No	360	21.69 ± 2.68	35.22 ± 4.51	24.96 ± 3.60	15.55 ± 2.73	97.43 ± 11.80

*t*			0.43	0.45	−0.34	−0.16	0.12
*P*			0.66	0.65	0.73	0.87	0.90
First choice	Yes	610	21.91 ± 2.57	35.71 ± 4.45	25.13 ± 3.67	15.72 ± 2.91	98.48 ± 11.82
	No	163	21.09 ± 2.90	33.75 ± 5.07	24.09 ± 3.82	14.82 ± 2.79	93.74 ± 12.95

*t*			3.55	4.87	3.18	3.56	4.46
*P*			<0.001	<0.001	0.002^*∗*^	<0.001	<0.001
Only child	Yes	262	22.09 ± 2.63	35.85 ± 4.55	25.46 ± 3.51	16.05 ± 2.75	99.45 ± 11.85
	No	511	21.56 ± 2.66	35.02 ± 4.68	24.63 ± 3.80	15.27 ± 2.96	96.47 ± 12.28

*t*			2.65	2.37	2.95	3.57	3.23
*P*			0.008^*∗*^	0.018^*∗*^	0.003^*∗*^	<0.001	0.001^*∗*^
Place of residence	Urban	483	21.94 ± 2.59	35.68 ± 4.60	25.19 ± 3.78	15.83 ± 2.91	98.64 ± 12.26
	Rural	290	21.40 ± 2.75	34.67 ± 4.68	24.44 ± 3.59	15.04 ± 2.85	95.55 ± 11.91

*t*			2.75	2.95	2.71	3.66	3.43
*P*			0.006^*∗*^	0.003^*∗*^	0.007^*∗*^	<0.001	0.001^*∗*^
Father's occupation	Nonmedical staff	749	21.72 ± 2.68	35.28 ± 4.67	24.88 ± 3.73	15.50 ± 2.93	97.38 ± 12.25
	Medical staff	24	22.42 ± 2.04	35.83 ± 4.23	25.83 ± 3.36	16.67 ± 2.10	100.75 ± 10.75

*F*			−1.27	−0.57	−1.23	−1.95	−1.33
*P*			0.21	0.57	0.22	0.05^*∗*^	0.18
Mother's occupation	Nonmedical staff	738	21.71 ± 2.68	35.26 ± 4.67	24.87 ± 3.73	15.48 ± 2.93	97.32 ± 12.24
	Medical staff	35	22.31 ± 2.26	36.20 ± 4.31	25.74 ± 3.60	16.66 ± 2.03	100.91 ± 11.16

*F*			−1.31	−1.17	−1.35	−2.35	−1.70
*P*			0.19	0.24	0.18	0.02^*∗*^	0.09
Father's education	Primary school or below	137	21.15 ± 2.90	34.66 ± 4.79	24.40 ± 3.66	15.01 ± 2.89	95.22 ± 12.46
	Junior high school	315	21.46 ± 2.59	34.81 ± 4.81	24.60 ± 3.68	15.20 ± 2.97	96.08 ± 12.22
	Senior high school	133	22.37 ± 2.68	35.93 ± 4.50	25.42 ± 3.96	15.67 ± 3.05	99.39 ± 12.37
	Vocational or junior college	108	21.96 ± 2.54	35.66 ± 4.39	24.69 ± 3.68	15.82 ± 2.51	98.14 ± 11.60
	Undergraduate or above	80	22.51 ± 2.25	36.79 ± 3.90	26.45 ± 3.21	17.09 ± 2.41	102.84 ± 10.27

*F*			6.50	4.42	5.43	8.47	7.18
*P*			<0.001	0.002^*∗*^	<0.001	<0.001	<0.001
Mother's education	Primary school or below		21.30 ± 2.78	34.74 ± 4.84	24.31 ± 3.96	14.75 ± 3.10	95.09 ± 12.72
	Junior high school		21.52 ± 2.66	34.70 ± 4.74	24.49 ± 3.60	15.23 ± 2.80	95.94 ± 11.95
	Senior high school		21.92 ± 2.25	35.80 ± 3.87	25.48 ± 3.35	15.84 ± 2.61	99.04 ± 10.51
	Vocational or junior college		22.45 ± 2.52	36.17 ± 4.50	25.53 ± 3.64	16.40 ± 2.59	100.55 ± 11.76
	Undergraduate or above		22.39 ± 2.73	37.05 ± 4.30	26.45 ± 3.51	17.07 ± 2.67	102.96 ± 11.79

*F*			5.35	6.01	7.01	13.45	9.49
*P*			<0.001	<0.001	<0.001	<0.001	<0.001
Family monthly income (RMB)	<3000	194	21.66 ± 2.76	35.64 ± 4.58	25.20 ± 3.56	15.40 ± 3.07	97.90 ± 12.24
	3000–6000	358	21.65 ± 2.65	34.96 ± 4.68	24.60 ± 3.70	15.35 ± 2.75	96.56 ± 12.15
	6000–10000	141	21.83 ± 2.60	35.33 ± 4.50	24.99 ± 3.76	15.79 ± 2.85	97.95 ± 11.47
	>10000	80	22.18 ± 2.61	35.95 ± 4.91	25.46 ± 4.10	16.18 ± 3.22	99.76 ± 13.44

*F*			0.97	1.54	1.81	2.27	1.76
*P*			0.41	0.20	0.15	0.08	0.15

The article "Research on the Relationship Model between Professional Identity and Life Meaning of Clinical Medical Freshmen based on Artificial Intelligence Medical Image Detection" was published in 2022. Journal: Contrast Media Mol Imaging.

**Table 5:** Results of the multivariate analysis of the professional identity of freshmen in clinical medicine (*n* = 773).

Variable	*B*	*S*‾*x*	*β*	*t*	*P*
Constant	56.90	4.24	—	13.41	<0.001

Nationality (Han nationality)					
Minority	1.57	0.92	0.05	1.69	0.09

First choice (yes)					
No	−3.26	0.87	−0.11	−3.74	<0.001

Only child (yes)					
No	−0.95	0.82	−0.04	−1.15	0.25

Place of residence (urban)					
Rural	−1.75	0.82	−0.07	−2.13	0.03^*∗*^

Father's occupation (nonmedical staff)					
Medical staff	0.19	2.36	0.00	0.08	0.94

Mother's occupation (nonmedical staff)					
Medical staff	0.34	2.02	0.01	0.17	0.87
Father's education	0.84	0.42	0.08	2.02	0.04^*∗*^
Mother's education	0.34	0.42	0.04	0.80	0.42

Family monthly income (RMB) (<3000)					
3000–6000	−2.15	0.89	−0.09	−2.40	0.02^*∗*^
6000–10000	−3.98	1.18	−0.13	−3.37	0.001^*∗*^
	−1.99	1.44	−0.05	−1.38	0.17

Meaning in life					
The presence of meaning in life	1.61	0.09	0.54	17.71	<0.001
The search for meaning in life	0.07	0.08	0.03	0.86	0.39

*Note.* ^*∗*^*P* < 0.05, *F* = 35.19, *P* < 0.001, *R*^2^ = 0.376, adjusted *R*^2^ = 0.365.

## Data Availability

The data underlying the results presented in the study are included within the manuscript.

## References

[1] Gleeson C. (2010). Education beyond competencies: a participative approach to professional development. *Medical Education*.

[2] Forouzadeh M., Kiani M., Bazmi S. (2018). Professionalism and its role in the formation of medical professional identity. *Medical Journal of the Islamic Republic of Iran*.

[3] Monrouxe L. V., Bullock A., Tseng H. M., Wells S. E. (2017). Association of professional identity, gender, team understanding, anxiety and workplace learning alignment with burnout in junior doctors: a longitudinal cohort study. *BMJ Open*.

[4] Ji L. K., Liu H. S., Li C. L. (2020). Boiled frogs in warm water: the influence mechanism of professional identity on college students’ depression. *Studies of Psychology and Behavior*.

[5] Zhang J. Y., Li D. (2016). College Students’ Professional identity and its relationship with achievement motivation and learning satisfaction. *China Journal of Health Psychology*.

[6] Zhang M., Li R. L. (2018). A study on the impact of college students’ professional identity on learning engagement: the mediating role of school belonging. *Heilongjiang Researches on Higher Education*.

[7] King L. A., Hicks J. A., Krull J. L., Gaiso A. K. D. (2006). Positive affect and the experience of meaning in life. *Journal of Personality and Social Psychology*.

[8] Lin L. (2021). Longitudinal associations of meaning in life and psychosocial adjustment to the COVID‐19 outbreak in China. *British Journal of Health Psychology*.

[9] Czekierda K., Banik A., Park C. L., Luszczynska A. (2017). Meaning in life and physical health: systematic review and meta-analysis. *Health Psychology Review*.

[10] Shahhosseini Z., Hamzehgardeshi Z., Marzband R., Azizi M. (2021). Meaning in life as a predictor of the general health among medical sciences students: a cross‐sectional study. *Nursing Open*.

The article "Research on the Relationship Model between Professional Identity and Life Meaning of Clinical Medical Freshmen based on Artificial Intelligence Medical Image Detection" was published in 2022. Journal: Contrast Media Mol Imaging.

[11] Qin P. B. (2009). The Characteristics and Correlation Study of College Students’ Specialty Identity.

[12] Wang M. C., Dai X. Y. (2008). Chinese Meaning in Life Questionnaire revised in college students and its reliability and validity test. *Chinese Journal of Clinical Psychology*.

[13] Kong W. H. (2019). *The Mediating Role of College Students’ Learning Self-Efficacy in the Relationship between Professional Identity and Learning Burnout*.

[14] Zhou Y., Liu X. W., Wu C. (2020). Status quo of major identity in undergraduates of a military medical university and its influencing factors. *Medical Journal of National Defending Forces in*.

[15] Tang M., Sun Y., Zhang K. (2022). Associated factors of professional identity among nursing undergraduates during COVID-19: a cross-sectional study. *International Journal of Nursing Science*.

[16] Boyle P. A., Buchman A. S., Bennett D. A. (2010). Purpose in life is associated with a reduced risk of incident disability among community-dwelling older persons. *American Journal of Geriatric Psychiatry*.

[17] Ji Y. L., Zang S. (2011). A study on the correlation between the meaning in life and positive perfectionism in medical students. *Health Vocational Education*.

[18] Ge Y., Shuai M. Q., Luo J., Wenger J. L., Lu C. Y. (2021). Associated effects of meaning in life and social adjustment among Chinese undergraduate students with left-behind experiences in the post-epidemic period. *Frontiers in Psychiatry*.

[19] Cho E.-H., Lee D.-G., Lee J. H., Bae B. H., Jeong S. M. (2014). Meaning in life and school adjustment: testing the mediating effects of problem-focused coping and self-acceptance. *Procedia-Social and Behavioral Sciences*.

[20] Halama P., DĚdov M. (2007). Meaning in life and hope as predictors of positive mental health: do they explain residual variance not predicted by personality traits?. *Studia Psychologica*.

[21] Cole S. W., Levine M. E., Arevalo J. M. G., Ma J., Weir D. R., Crimmins E. M. (2015). Loneliness, eudaimonia, and the human conserved transcriptional response to adversity. *Psychoneuroendocrinology*.

[22] Hicks J. A., Schlegel R. J., King L. A. (2010). Social threats, happiness, and the dynamics of meaning in life judgments. *Personality and Social Psychology Bulletin*.

[23] Bamonti P., Lombardi S., Duberstein P. R. V. (2016). Spirituality attenuates the association between depression symptom severity and meaning in life. *Aging & Mental Health*.

[24] Huai D. D., Cao G. F., Sun X. (2020). A study on the impact of Life Meaning of rural-oriented medical students on professional identity. *Chinese Health Service Management*.

The article "Research on the Relationship Model between Professional Identity and Life Meaning of Clinical Medical Freshmen based on Artificial Intelligence Medical Image Detection" was published in 2022. Journal: Contrast Media Mol Imaging.

[25] Zhu H. T., Yao X. X. (2015). The meaning in life and depression in college freshmen: interaction and mediation effects. *Psychological Development and Education*.

[26] Zhu J. C., Wang X. Q. (2017). The relationship between professional identity and suicidal ideation in normal students: the mediating role of depression and its gender differences. *Psychological Development and Education*.

[27] Wang L., Yang Y., Zhu J. (2019). Professional identity and mental health of rural-oriented tuition-waived medical students in Anhui Province, China. *BMC Medical Education*.

[28] Khan R., Apramian T., Kang J. H., Gustafson J., Sibbald S. (2020). Demographic and socioeconomic characteristics of Canadian medical students: a cross-sectional study. *BMC Medical Education*.

[29] Sapkota B. P., Amatya A. (2015). What factors influence the choice of urban or rural location for future practice of Nepalese medical students? A cross-sectional descriptive study. *Human Resources for Health*.

